The article "A Cohort Study of Surgical Indexes, Postoperative Complications, Recovery Speed, and Prognosis of Stanford Type A Aortic Dissection Compared with Traditional Sun's Operation" was retracted in 2023. Reasons: unreliable results or conclusions; concerns about the data; concerns about the peer review; concerns about the citations.

# A Cohort Study of Surgical Indexes, Postoperative Complications, Recovery Speed, and Prognosis of Stanford Type A Aortic Dissection Compared with Traditional Sun's Operation

**DOI:** 10.1155/2022/9516922

**Published:** 2022-11-11

**Authors:** Yiqing Feng, Jianli Ren, Yihe Zhang, Hu Liu, Xingxing Ma, Jing Guo

**Affiliations:** Cardiovascular Center, Affiliated Hospital of Yan'an University, Yan'an 716000, China

## Abstract

**Objective:**

The objective is to explore the surgical index, postoperative complications, recovery speed, and prognosis of Stanford type A aortic dissection (AD) compared with traditional 'Sun's operation.

**Methods:**

One hundred patients with Stanford type A AD treated from February 2018 to February 2021 were enrolled in our hospital. Patients were randomly divided into control and research group. The former group underwent traditional Sun's surgery, and the latter group underwent combined debranching surgery. The general data, surgical indexes, total amount of blood transfusion, renal function 72 hours after operation, postoperative indexes during hospitalization, and follow-up results after discharge were compared between the two groups.

**Results:**

The CPB time, ACC time, operation time, and postoperative total drainage volume of the study group were all lower than those of the control group, and the intraoperative urine volume of the study group was higher than that of the control group (*P* < 0.05). The total amount of RBC infused in the study group was higher than that in the control group, while the total amount of PLT, cryoprecipitate, and plasma infusion in the study group was lower than that in the control group (*P* < 0.05). At 72 hours after operation, BUN, Scr, and UA in the study group were significantly lower than those in the control group (*P* < 0.05). The number of the secondary intubation, hemodialysis, neurological complications, and deaths in the study group was significantly lower than that in the control group (*P* < 0.05).

**Conclusion:**

Both Sun's operation and branch removal are more effective treatment methods, and the two different surgical methods have different indications, advantages, and disadvantages, so different surgical methods can be chosen according to different conditions for Stanford AD. The possible postoperative complications should be comprehensively analyzed in the clinical work in order to reduce the occurrence of postoperative complications and improve the cure rate.

## 1. Introduction

Aortic dissection (AD) is a kind of aortic syndrome, which is known for its high risk and high mortality and is often called a ticking time bomb [1]. The first symptoms of AD are usually severe pain in the chest or back. It has the characteristics of acute onset, critical condition, and rapid progress. There is currently no effective method for early diagnosis [1, 2]. According to a 20-year statistical result of AD published by M. A. A. Jawad in 2020 [2], the overall incidence of AD in the population is 4.4 cases/100,000 person-years. Due to the acute onset, rapid progression, high misdiagnosis rate, and critical condition, if patients are not treated in time, the mortality rate of acute AD in the early stage (within 48 hours) is as high as 50%, and a large number of patients have died before receiving treatment. Surgery is the only way to save the lives of AD patients. A large-scale study in 2005 shows that surgical intervention can reduce the mortality rate of patients with acute AD from 90% to 30% within 1 month and then experience 10 years of development [3]. AD is more common in the elderly with coronary heart disease and hypertension, usually the severe sudden pain in the front chest or back is the first symptom, it has the characteristics of sudden onset, dangerous condition, and rapid progress. Once the disease occurs, the mortality rate can be as high as 54% and 76% within 6 hours and 24 hours without treatment [4, 5].

In order to help the better treatment of AD, many methods have been developed to classify AD. The first is DeBakey classification, that is to say, the primary breach of the dissection was located in the ascending aorta (AA) or arch, and it could gradually involve the abdominal aorta from the AA to the distal end, which was type 1 [6]. The primary rupture and the extent of involvement were limited to type 2 in the AA, and the primary rupture was located at the distal end of the opening of the left subclavian artery and could continue to be involved distally, even reaching the abdominal aorta in type 3 [6]. In addition, there is the Stanford classification, that is, as long as the AD involves the AA, it is type A. The left subclavian artery orifice is far involved, and the AA is not involved; it is type A [7]. In order to help surgeons better grasp the surgical indications and surgical methods of acute AD, Sun Lizhong and others in Beijing Anzhen Hospital put forward a detailed classification of Stanford classification [8]. According to the different conditions of aortic root involvement, type A dissection was assigned into three types: A1, A2, and A3, that is, A1 was normal in aortic sinus and A2 was slightly involved in aortic sinus. Those with severe aortic valve involvement are called type A3. In addition, according to the involvement of the aortic arch, it is assigned to C type and S type. Due to the inherent sudden onset and dangerous characteristics of acute type A AD, it is difficult to treat patients [9]. According to the clinical data of major heart centers across the country, the effect of simple conservative treatment and interventional therapy for type A aortic dissection is poor, Sun's surgical treatment (that is, total arch replacement + stent trunk technique) and later developed debranching technique combined with thoracic aortic stent implantation are more effective, which can reduce the mortality in patients to the greatest extent and enhance the survival rate. From the point of view of the type of operation, Sun's operation belongs to open surgery, while the debranching technique combined with thoracic aortic stent implantation is a hybrid technique of open surgery combined with stent intervention. However, how to choose the two surgical methods, their respective advantages and disadvantages, and the best surgical indications need to be further studied and discussed [10]. Dissection can involve all or parts of the abdominal aorta from the AA to the distal end, and the risk of rupture under the impact of high pressure blood flow is greatly increased. Therefore, it is particularly important to choose the most appropriate treatment to reduce the short-term and long-term mortality in patients. Based on this, the purpose of this study is to explore the surgical index, postoperative complications, recovery speed, and prognosis of Stanford type A AD compared with the traditional Sun's operation.

## 2. Patients and Methods

### 2.1. Normal Information

One hundred patients with Stanford type A AD (thoracic aorta dilation) treated from February 2018 to February 2021 were enrolled in our hospital. Patients were randomly divided into the control and research group. The former group underwent traditional Sun's surgery, and the latter group underwent combined debranching surgery. In the control group, the age was 54–75 (63.49 ± 10.31) years and male/female was 26/24; in the research group, the age was 51–77 (63.59 ± 10.64) years and male/female was 27/23. There exhibited no statistical significance in the general data (see Table 1). This study was permitted by the Medical Ethics Association of our hospital (number: YAU-20180001), and all patients noticed informed consent.

The selection criteria are as follows: (1) all patients were diagnosed as Stanford type A AD by CTA and echocardiography before operation; (2) the age was ≥30 years and ≤80 years; (3) all patients and their immediate family members had signed preoperative informed consent; and (4) there were no operative contraindications.

The exclusion criteria are as follows: (1) the patient is a pregnant or lactating woman; (2) the patient has respiratory insufficiency before operation; (3) the patient has chronic renal dysfunction or has been treated with hemodialysis; (4) the patient is allergic to contrast media and anesthetics; (5) the patient is in poor physical condition and cannot tolerate any surgical treatment; and (6) the patient has severe heart disease (such as ventricular arrhythmia and congestive heart failure).

In terms of the general data, there exhibited no significant difference in age, sex, left ventricular diameter, LVEF, diabetes, hypertension, and Marfan syndrome (*P* > 0.05). All the data results are indicated in Table 1.

### 2.2. Treatment Methods

The doctors who performed the operation in this study were all in the same team. The patients in the control group received traditional Sun's surgery. Sun's surgical method is as follows: the sternum is split longitudinally, the brachiocephalic artery, aortic arch and axillary artery are completely separated, the atrial venous cannula is inserted, and the right subclavian artery is inserted into the arterial canal. Meanwhile, the right superior pulmonary vein was inserted into the left atrial drainage tube to establish cardiopulmonary bypass. Meanwhile, the patient's body temperature was gradually reduced, and ice shavings can be used to cool the heart surface. When ventricular fibrillation (VF) occurs, the AA is occluded. Of note, the proximal aorta is cut open and cardioplegia is perfused through bilateral coronary openings. Carefully examine the scope and severity of aortic root involvement, and then carry out the corresponding treatment according to different types of lesions. At present, these are the following main methods: coronary artery bypass grafting is feasible when the coronary artery is seriously involved, valve replacement is feasible when the lesion is severely involving the aortic valve, and Bentall and David procedures can be performed according to the condition of the root disease in order to completely relieve the root lesion. When the temperature of nasopharynx dropped to 18–20°C, the left common carotid artery (LCCA), left subclavian artery (LSCA), and innominate artery (IA) were blocked, respectively, and then circulatory arrest and unilateral cerebral perfusion were performed in the lower body. To begin to deal with the distal end of the aorta, it is necessary to insert the stent-like artificial vessel into the true lumen of the descending aorta (DA), anastomose it with the aortic wall and the distal end of the quadruple artificial vessel, exhaust and restore the blood supply of the lower body, and then anastomose the collateral branches of the aortic arch with the branches of the quadrilateral vessel. Finally, stop after rewarming, ultrafiltration of blood, autologous blood transfusion, routine postoperative hemostasis and chest closure, and return to the intensive care unit.

The research group received debranching combined operation and debranching hybrid operation: longitudinal split sternotomy, full dissociation of brachiocephalic artery, aortic arch and axillary artery, insertion of the vein tube in the atrium and arterial tube in the right subclavian artery. Meanwhile, the right superior pulmonary vein was inserted into the left atrial drainage tube to establish cardiopulmonary bypass, and the patient's body temperature was gradually reduced. Ice shavings can be adopted to cool the heart surface. When VF occurs, the AA should be blocked. Of note, the proximal aorta should be cut open and cardioplegia is perfused through bilateral coronary openings. Carefully examine the scope and severity of aortic root involvement, and then carry out the corresponding treatment according to different types of lesions. At present, these are the following main methods: coronary artery bypass grafting is feasible when the coronary artery is seriously involved, valve replacement is feasible when the lesion is severely involving the aortic valve, and Bentall and David procedures can be performed according to the condition of the root disease in order to completely relieve the root lesion. Waiting for the temperature of nasopharynx to drop to moderate hypothermia (25°C∼28°C), the AA was replaced and anastomosed by four-bifurcated blood vessels, then the aortic clamp was released and began to rewarm, at this time, the brachiocephalic artery was anastomosed with the bifurcated artificial vascular branches. After all the blood vessels were anastomosed and the rewarming was satisfactory, the machine began to stop. Then, with the assistance of DSA and interventional delivery device, the thoracic aortic stent was sent to the designated position of the aorta, and the appropriate position was determined by angiography to release it and ensure that the proximal end and distal end of the stent were anchored at the distal end and DA end of the artificial vessel, respectively. DSA angiography was performed again after operation to confirm the fixation of the covered stent and whether there was internal leakage. If the anchorage position of the stent is good and there is no internal leakage, withdraw the interventional catheter. Finally, the blood was treated by ultrafiltration, autologous blood transfusion, routine postoperative hemostasis and chest closure, and returned to the intensive care unit.

### 2.3. Observation Index

#### 2.3.1. General Information

The age, sex, left ventricular diameter, LVEF, diabetes, hypertension, and the Marfan syndrome were counted.

#### 2.3.2. Operation Index

The CPB time, ACC time, operation time, total postoperative drainage, and intraoperative urine volume were calculated.

#### 2.3.3. Total Blood Transfusion of Various Components during Operation

The total amount of RBC infusion, PLT, cryoprecipitation, and plasma transfusion were calculated.

#### 2.3.4. Renal Function

The renal function (BUN, Scr, UA) was calculated 72 hours after operation.

#### 2.3.5. Postoperative Index during Hospitalization

The number of twice intubation, hemodialysis, neurological complications, and deaths after 1 week after operation was calculated.

#### 2.3.6. Postoperative Follow-Up

All patients were followed up for 1 year after discharge by telephone or in-hospital reexamination; the follow-up indicators were the occurrence of postoperative complications and the number of deaths.

### 2.4. Statistical Analysis

SPSS 23.0 statistical software was adopted to process the data. The measurement data were presented as ($\bar{x}$ ± *s*). The group-designed *t*-test was adopted for the comparison, and the analysis of variance was adopted for the comparison between multiple groups. Dunnet'stest was adopted for comparison with the control group. The counting data were presented in the number of cases and percentage, *χ*^2^ test was adopted for comparison between the groups, and bilateral test was employed for all statistical tests.

## 3. Results

### 3.1. Comparison of Surgical Indexes

The CPB time, ACC time, operation time, and postoperative total drainage volume of the research group were all lower than those of the control group, and the intraoperative urine volume of the research group was higher than that of the control group (*P* < 0.05). All the data results are indicated in Table 2.

### 3.2. Comparison of the Total Amount of Blood Components Infused during Operation

With regard to the total amount of various components of blood transfusion during operation, the total amount of RBC infusion in the research group was higher than that in the control group, while the total amount of PLT, cryoprecipitation, and plasma transfusion in the research group was lower than that in the control group (*P* < 0.05). All the data results are indicated in Table 3.

### 3.3. Comparison of Renal Function at 72 hours after Operation

BUN, Scr, and UA in the research group at 72 hours after operation were lower than those in the control group (*P* < 0.05). All the data results are indicated in Table 4.

### 3.4. Comparison of Postoperative Indexes during Hospitalization

Regarding the postoperative indexes during hospitalization, the incidence of the secondary intubation, hemodialysis, neurological complications, and the number of deaths one week after operation in the research group were lower than those in the control group (*P* < 0.05). All the data results are indicated in Figure 1.

### 3.5. Comparison of Follow-Up Results after Discharge

With regard to the follow-up results after discharge, the number of deaths, the incidence of internal leakage, the number of deaths from pulmonary infection, the number of deaths from cerebral infarction, and the number of deaths from heart failure in the research group were lower than those in the control group (*P* < 0.05). All the data results are indicated in Figure 2.

## 4. Discussion

The purpose of this study is to explore the surgical index, postoperative complications, recovery speed, and prognosis of Stanford type A AD compared with the traditional Sun's operation. Aortic dissection (AD) is a kind of acute aortic disease with high mortality [11, 12]. The incidence rate of AD is increasing year-by-year, and the ratio of male to female is nearly 3 : 2 [13]. According to 2016 data from the world's largest International Registry of Acute AD (IRAD), the early mortality rate of patients with acute AD is still 17%–26%, which means that under existing medical methods, even after the most complex surgical treatment, patients have a very high risk of death, so the strategy optimization of each treatment link cannot be underestimated [14]. The pathological manifestations are aortic intima tear, intima rupture, aortic nutrient vessel rupture, and media hemorrhage caused by many reasons. Due to the destruction of membrane structural integrity or intima-media vascular hemorrhage, blood flow cannot be discharged from the intermembrane, but it accumulates to form a dissecting hematoma and expand around, gradually peels off the aortic intima and media, and separates the aortic lumen into a true lumen and a false lumen. It eventually leads to dilation or rupture of the aorta [15]. Studies have indicated that the average age of people with AD is 63 years, and men are more likely to develop the disease than women, with a male-to-female ratio of nearly 3 : 2 [16]. It is worth noting that the incidence of AD in China not only gradually developed from the initial middle-aged and elderly to adolescents, but also increased remarkably [17]. Due to the great differences in clinical manifestations, such as chest pain, nerve defect, or syncope, the diagnosis of the disease becomes more difficult and the possibility of missed diagnosis and misdiagnosis increases [18]. Meanwhile, it is also a kind of acute aortic disease with a high mortality rate [19, 20]. Once this disease occurs, the mortality rate can be as high as 54% and 76% within 6 hours and 24 hours, respectively [21]. The main causes of death are a series of complications caused by continuous tearing of dissection and enlargement of false lumen, such as acute hemorrhagic shock, acute heart failure caused by aortic valve or coronary artery involvement, acute renal failure caused by renal artery involvement, and rapid retroperitoneal or mediastinal hemorrhage. Acute pericardial tamponade can be caused by rupture of pericardial cavity or thoracic cavity of AD. Mesenteric ischemia can be caused by various causes [22]. After years of continuous development and continuous improvement of the medical level, the treatment methods for this disease are gradually increasing, but generally speaking, it mainly includes nonoperative treatment and surgical treatment, especially for type A AD. Surgical treatment is still the most important treatment for this disease [23].

There are many different views on the pathogenesis of AD, but its exact mechanism is still unclear. The first is the mechanism of immune inflammation; when AD occurs, a large number of macrophages infiltrate in the vascular wall, which on the one hand causes inflammatory reaction, and on the other hand, it can degrade elastic fibers through the release of matrix metalloproteinases, which destroys the middle structure of the aortic wall and leads to the formation of AD [24]. Studies have found that neutrophils also attach importance to the pathogenesis of AD. Lesion-infiltrating neutrophils secrete matrix metalloproteinase 9 and IL-6 to degrade elastic fibers, thereby accelerating the rupture of AD [25]. IL1 *β* can promote the secretion of matrix metalloproteinases by smooth muscle cells and macrophages, which may be related to the phosphorylation of p38 pathway, which destroys the middle structure of the aortic wall and leads to AD [26]. The second is genetic factors, such as the Marfan syndrome and aortic valve bivalvular malformation. Marfan syndrome is an autosomal dominant genetic disease involving connective tissue, which can involve cardiovascular, bone, and other organs, especially when the cardiovascular system is involved in time, it can lead to necrosis, rupture, or deformity of the middle structure of the aortic wall. Intimal rupture can be easily caused by the lack of media support structure [27]. Aortic valvular malformation is not only an autosomal dominant hereditary disease, but also a congenital heart disease. Patients with this disease are often accompanied by dilated AA, which increases the risk of AD by a factor of 9 [28]. The third is oxidative stress, which means that when the body is stimulated by external harmful factors or some cells in the body need to be removed, there are too many oxidation products in the body and the ability to remove oxidation products is inadequate. As a result, the balance between oxidation and antioxidation is broken, which leads to damage to the tissue structure of the body. It is considered that the morphological basis of AD is the destruction of elastic fibers in the middle structure of the aortic wall [29]. During oxidative stress, the binding of elastin and fibulin5 is inhibited by reactive oxygen species, which destroys the elastic fibers of the middle structure of the aortic wall, resulting in the fragility of the aortic wall, and intimal tearing and dissection is more likely to occur under the impact of high pressure blood flow in the aortic lumen. The fourth is atherosclerosis, the pathological process of this disease is the deposition of lipids in the intima of the artery to form lipid lines, the formation of fibrous plaques, and then the formation of atherosclerotic plaques, resulting in secondary changes and in wall thickening and lumen stenosis [30]. In the process of atherosclerosis, the smooth muscle and elastic fibers of the middle layer of the arterial wall will be broken and destroyed, and a relatively weak area will appear. Under the impact of high pressure blood flow in the aortic lumen, the intima will be torn, and the blood will enter from the intimal rupture to the middle layer, forming AD [31]. In addition, atherosclerosis can also cause the production of oxidized low density lipoprotein, which in turn leads to the expression of cytokines and induces the release of leukocytes to the inflammatory site through adhesion, aggregation, migration, and chemotaxis, leading to the production and development of AD [32]. Finally, angiotensin II, on the one hand, can damage the intimal structure of the artery by causing an increase in blood pressure, resulting in a rupture of the intima under the impact of blood flow, leading to the formation of dissection. On the other hand, angiotensin II can induce apoptosis of vascular endothelial cells, and its mechanism may be related to monocyte chemoattractant protein 1 expressed by vascular endothelium [33]. Once vascular endothelial cells are injured by apoptosis, it will greatly increase the probability of arterial intimal rupture and dissection.

It is well known that Sun's operation is the first main treatment for type A AD, which can be solved thoroughly by ascending aortic replacement + total arch replacement + stent elephant trunk technique. Prevent the death of patients caused by the rupture of dissection [34]. However, this kind of operation requires artificial vascular replacement of the arch, which requires that the operation should be carried out under the condition of deep hypothermic circulatory arrest and selective cerebral perfusion, and deep hypothermic circulatory arrest has a great impact on the function of various organs of the whole body, especially the perfusion of the nervous system and kidney, which can easily bring about a series of complications and indirectly affect the effect of the whole operation. Therefore, the protection of various organs should be fully considered when Sun's operation is carried out, which increases the difficulty of the operation. Later, with the continuous development of the intracavitary technology, stent implantation was gradually applied to the treatment of type A AD, the arch was treated with debranching technique, and then thoracic aortic stent implantation was performed on the distal DA, which is also called compound technique or hybrid technique [35–37]. It does not need deep hypothermic circulatory arrest, and the treatment of distal DA does not need the assistance of cardiopulmonary bypass, which relatively shortens the auxiliary time of cardiopulmonary bypass. Furthermore, it reduces the incidence of postoperative complications and mortality caused by deep hypothermic circulatory arrest and long-term cardiopulmonary bypass [38, 39]. However, the debranching technique combined with distal stent implantation also has certain defects, such as the high incidence of endoleak caused by stent implantation and the long-term decay of the stent. Therefore, even for debranching combined surgery, continuous improvement is needed to gradually reduce surgical complications. But meanwhile, we also need to note that the development from Sun's surgery to branch removal is undoubtedly a great progress in the field of large blood vessels, which provides a variety of options for the treatment of patients with type A AD [40]. This study still has some shortcomings. Firstly, the quality of this study is limited due to the small sample size we included in the study. Secondly, this research is a single-center study and our findings are subjected to some degree of bias. Therefore, our results may differ from those of large-scale multicenter studies from other academic institutes. We considered that the aortic diameters were homogenous, there may still have been unavoidable selection bias from unknown factors affecting proximal aorta dimensions. This research is still clinically significant and further in-depth investigations will be carried out in the future.

In summary, both Sun's operation and branch removal are more effective treatment methods, and the two different surgical methods have different indications, advantages, and disadvantages, so different surgical methods can be chosen according to different conditions for Stanford AD. The possible postoperative complications should be comprehensively analyzed in the clinical work in order to reduce the occurrence of postoperative complications and improve the cure rate.

## Figures and Tables

**Figure 1:** Comparison of postoperative indexes during hospitalization between the two groups.

**Figure 2:** Comparison of follow-up results after discharge between the two groups.

**Table 1:** Comparison of general data of the two groups of patients.

Groups	*N*	Age	Male/female	Diabetes	Marfan syndrome	High blood pressure	Left ventricular diameter	LVEF (%)
Control group	50	63.49 ± 10.31	26/24	14 (28.00)	10 (20.00)	41 (82.00)	54.69 ± 5.53	50.91 ± 5.78
Research group	50	63.59 ± 10.64	27/23	13 (26.00)	11 (22.00)	40 (80.00)	54.95 ± 5.47	50.44 ± 5.57
*t*/*χ*^2^ value		0.047	0.135	0.124	0.113	0.078	0.236	0.414
*P* value		>0.05	>0.05	>0.05	>0.05	>0.05	>0.05	>0.05

**Table 2:** Comparison of surgical indexes between the two groups [$\bar{x}$ ± *s*].

Groups	*N*	CPB time (min)	ACC time (min)	Operation time (h)	Intraoperative urine volume (ml)	Total postoperative drainage (ml)
Control group	50	245.93 ± 53.31	178.49 ± 34.46	8.49 ± 1.44	707.84 ± 54.77	1564.95 ± 57.44
Research group	50	110.93 ± 45.64	137.38 ± 34.23	5.35 ± 1.53	1304.59 ± 23.55	1185.72 ± 53.77
*t* value		**13.602**	**5.984**	**10.567**	**70.777**	**34.081**
*P* value		<**0.05**	<**0.05**	<**0.05**	<**0.05**	<**0.05**

**Table 3:** Comparison of the total amount of various components of blood transfusion between the two groups [$\bar{x}$ ± *s*].

Groups	*N*	RBC (u)	PLT (u)	Cold precipitation (u)	Plasma (ml)
Control group	50	11.55 ± 3.53	2.46 ± 1.43	6.73 ± 3.31	3135.66 ± 346.34
Research group	50	13.53 ± 3.78	1.48 ± 0.78	4.51 ± 2.45	2243.85 ± 374.42
*t* value		**2.707**	**4.254**	**3.811**	**12.363**
*P* value		<0.05	<0.05	<0.05	<0.05

**Table 4:** Comparison of the renal function between the two groups at 72 hours after operation [$\bar{x}$ ± *s*].

Groups	*N*	BUN (mmol/L)	Scr (umol/L)	UA (umol/L)
Control group	50	10.94 ± 3.45	110.59 ± 24.65	356.24 ± 59.55
Research group	50	6.13 ± 0.75	85.39 ± 13.56	321.67 ± 64.32
*t* value		**9.633**	**6.333**	**2.788**
*P* value		<**0.05**	<**0.05**	<**0.05**

## Data Availability

The datasets used and analyzed during the current study are available from the corresponding author upon reasonable request.
